# A Core Drug Discovery Framework from Large-Scale Literature for Cold Pathogenic Disease Treatment in Traditional Chinese Medicine

**DOI:** 10.1155/2021/9930543

**Published:** 2021-08-04

**Authors:** Yun Zhang, Yongguo Liu, Jiajing Zhu, Zhi Chen, Dongxiao Li, Yonghua Xiao, Xiaofeng Liu, Shuangqing Zhai

**Affiliations:** ^1^Knowledge and Data Engineering Laboratory of Chinese Medicine, School of Information and Software Engineering, University of Electronic Science and Technology of China, Chengdu 610054, China; ^2^Sichuan Academy of Chinese Medical Sciences, Chengdu 610041, China; ^3^Dongzhimen Hospital, Beijing University of Chinese Medicine, Beijing 100700, China; ^4^School of Basic Medical Science, Beijing University of Chinese Medicine, Beijing 100029, China

## Abstract

Cold pathogenic disease is a widespread disease in traditional Chinese medicine, which includes influenza and respiratory infection associated with high incidence and mortality. Discovering effective core drugs in Chinese medicine prescriptions for treating the disease and reducing patients' symptoms has attracted great interest. In this paper, we explore the core drugs for curing various syndromes of cold pathogenic disease from large-scale literature. We propose a core drug discovery framework incorporating word embedding and community detection algorithms, which contains three parts: disease corpus construction, drug network generation, and core drug discovery. First, disease corpus is established by collecting and preprocessing large-scale literature about the Chinese medicine treatment of cold pathogenic disease from China National Knowledge Infrastructure. Second, we adopt the Chinese word embedding model SSP2VEC for mining the drug implication implied in the literature; then, a drug network is established by the semantic similarity among drugs. Third, the community detection method COPRA based on label propagation is adopted to reveal drug communities and identify core drugs in the drug network. We compute the community size, closeness centrality, and degree distributions of the drug network to analyse the patterns of core drugs. We acquire 4681 literature from China national knowledge infrastructure. Twelve significant drug communities are discovered, in which the top-10 drugs in every drug community are recognized as core drugs with high accuracy, and four classical prescriptions for treating different syndromes of cold pathogenic disease are discovered. The proposed framework can identify effective core drugs for curing cold pathogenic disease, and the research can help doctors to verify the compatibility laws of Chinese medicine prescriptions.

## 1. Introduction

Cold pathogenic disease (CPD, 中医伤寒) is the general term for exogenous febrile diseases in traditional Chinese medicine (TCM), which are a class of diseases appearing with fever as the main clinical symptom caused by feeling pathogenic factors and six climatic exopathogens (wind, cold, heat, wet, dryness, and fire, 六种外感病邪) in TCM [1–3]. With the development of CPD, different stages (Tai-Yang, Yang-Ming, Shao-Yang, Tai-Yin, Shao-Yin, and Jue-Yin syndromes) will occur coming from the summary of various symptoms when humans feel pathogenic factors based on the basic theories of TCM [1]. CPD has the characteristics of rapid onset, fast spread, and obvious fever with cough and headache [2, 3], which have similar early symptoms with COVID-19 [4]. As a frequent occurrence disease, CPD often results in the onset and aggravation of internal injury and severe acute diseases [5–7]. The external cause of CPD is mainly seasonal pathogens, which can be summarized as the four types of wind-cold, warm-heat, damp-heat, and epidemic diseases in TCM, and its internal cause is the low immunity of humans [3, 5].

CPD contains some typical illnesses, such as influenza and respiratory infection in Western medicine [8, 9]. Influenza circulates in the global and can influence the people in all age groups, which leads to a severe public health problem. The 3,000,000 to 5,000,000 serious illnesses and about 250,000 to 500,000 deaths every year are related to influenza [10, 11]. Influenza outbreak could bring about huge loss. The 1918 Spanish flu pandemic brought about twenty to fifty million deaths reportedly [4]. The 1957 Asia flu and 1968 Hong Kong flu caused one million deaths [11]. The influenza in the early stage will causes the symptoms of fever, cough, headache, stuffy nose, and runny nose, which may damage lung function and threat human life when it becomes severe and concurrences with other diseases [8]. For the prevention and treatment of CPD, Chinese medicine has accumulated experience in thousands of years to form unique treatment and achieve clinical effects [12, 13]. For example, classic prescriptions Gui-Zhi decoction [14] and Si-Jun-Zi decoction [15] are formed.

TCM has diverse therapies, such as medicinal prescription, medicinal wine, medicinal diet, acupuncture, scraping, and cupping [16, 17]. Among these therapies, medicinal prescription is used frequently, which has lots of features, such as compatibility composition, taboo, efficacy, and usage [17, 18]. The compatibility composition of medicinal prescription can reflect the rationality of drug combinations to determine the effectiveness of prescriptions for treating different syndromes and diseases [16, 17]. “Jun-Chen-Zuo-Shi” composition principle, also called as “sovereign-minister-assistant-courier” composition principle, is a major form of compatibility composition in TCM [19, 20], in which the drugs acting as “Jun” or “Chen” play the key therapeutic effect, while other drugs serving as “Zuo” or “Shi” play the supporting function in certain prescriptions [20]. Thus, we can consider “Jun” and “Chen” drugs as core drugs in medicinal prescriptions [21, 22]. There are large-scale electronic medical records and literature recording TCM prescriptions; however, they do not record core drug information. Core drug discovery is important for uncovering the correlation between prescriptions and syndromes to verify the compatibility law of TCM prescriptions and helping young doctors and learners to study the essence of TCM prescriptions [23]. According to the discovered core drugs for treating different syndromes of CPD, doctors can optimize compatibility combinations and find more effective prescriptions, which is helpful for accurate medication.

Researchers mainly explored the problem of core drug discovery by manual literature analysis [24, 25], medical experiment [20, 26], and data mining [21–23, 27, 28]. At the early stage, researchers searched the relevant books about the treatment of a specific syndrome in TCM, analysed the possible relations between drugs and syndromes, and determined core drugs based on frequent relations, whose efficiency is low [24, 25]. Medical experiments can be classified as clinical and pharmacology experiments [20, 26]. In the former, the effect of different drug combinations is measured on patients (volunteers) to discover drugs with good outcomes; then, they are considered as core drugs [26]. In the latter, pharmacology criteria are defined to evaluate the scores of different ingredients of TCM prescriptions; then, they regarded the drugs with high score ingredients as core drugs [20]. However, testing all drug compatibility and ingredients in the experimental manner is difficult. Data mining methods analysed the compatibility rules and core drugs of TCM prescriptions in medical records by computing the frequency and co-occurrence relations of drugs in TCM prescriptions [27, 28], which mainly concentrate on analysing medical records and can handle large-scale data [29, 30]. However, they cannot comprehend the implication of drugs in these records. For instance, Chinese drug *milkvetch root* has a lot of characteristics, such as efficacy, dosage, and taboo, but these methods cannot capture these features from the texts of this Chinese word because they only consider the drug as a text, such as an English letter. Meanwhile, there are rich literature containing medical knowledge besides medical records [22]. However, there are few research studies to discover core drugs from literature, which may be caused by the difficulty of data processing. The medical records are structured texts, but the literature text is unstructured, where syndrome, prescription, and drug are distributed in full text unevenly. Some researchers analysed few TCM literature to mine specific treatment patterns existing in TCM prescription [28, 31], but also consider the drug as a text. Zhang et al. [22] adopted the semantic analysis method to extract the drug semantic in literature and mine the core drugs for treating chronic glomerulonephritis.

In order to enhance the efficiency of literature analysis and understand drug implication in literature, we introduce word embedding [32] and community detection [33] to handle the unstructured text in literature and identify core drugs for curing different syndromes of CPD. In this paper, we design a core drug discovery framework (CDDF) for detecting core drugs for treating CPD from literature, which contains three parts: disease corpus construction, drug network generation, and core drug discovery. In the first stage, large-scale relevant literature about the TCM treatment of CPD is searched in China National Knowledge Infrastructure (CNKI) and preprocessed automatically to build disease corpus. In the second stage, we adopt Chinese word embedding model SSP2VEC, which is proposed in [32] by us, and it considers the inner-character attributes (stroke, structure, and pinyin) and their relevance to mine the meanings of drugs in literature and expresses drugs as semantic vectors for calculating drug similarity and building the drug network. In the third stage, drug communities and core drugs are discovered in the drug network by community detection algorithm COPRA [33], in which the communities and important nodes are modelled as drug communities and core drugs. In order to research the drug network further, we compute its community size, closeness centrality, and degree distributions to analyse the patterns of core drugs. Experiment results show that CDDF reveals 12 major drug communities where drugs have similar efficacy in each community and 4 classical TCM prescriptions for treating CPD. Meanwhile, top-10 drugs with most correct core drugs for treating CPD are found in each drug community.

## 2. Related Work

Many research studies for discovering core drugs have been published, which can be divided into three types: manual literature analysis [24, 25], medical experiment [20, 26], and data mining [21–23, 27, 28]. Here, we briefly introduce the related work.

For manual analysis, researchers usually artificially searched some literatures about the TCM treatment of a specific syndrome, extracted TCM prescriptions, and detected core drugs. Lin et al. [24] extracted the acupuncture prescriptions from authority TCM books, such as Huang-Di-Nei-Jing, for mining “Jun-Chen-Zuo-Shi” drugs. Lin and Huang [25] analysed the principle of “Jun-Chen-Zuo-Shi” according to Shen-Nong-Ben-Cao-Jing.

Medical experiments include pharmacology and clinical trials, in which investigators mined effective drug ingredients or combinations of TCM prescriptions for discovering the core drugs to cure a certain syndrome, respectively. A network pharmacology approach is used for identifying the “Jun-Chen-Zuo-Shi” drugs in Qi-Shen-Yi-Qi prescription to cure myocardial ischemia [20]. The protein-protein interactions and disease-associated genes are integrated to establish an organism disturbed network. Based on the network, the network recovery index (NRI) is proposed for evaluating the curative effect of Qi-Shen-Yi-Qi prescription and its ingredients. As a result, the prescription gets 864.48 NRI score, which is higher than a single drug. When these drugs form prescription, they obtain better effect than a single drug. In addition, the NRI scores of *danshen root* and *milkvetch root* are 734.31 and 680.27, respectively; thus, they are considered as core drugs. Yan et al. [26] designed a protocol to conduct a triple-blind and randomized clinical trial to discover core drugs by association rules for curing primary insomnia.

For data mining methods, most researchers mainly analysed medical records to mine drug frequency and their co-occurrence relationships among drugs in prescriptions for discovering core drugs. Combining interdisciplinary technology is the trend for discovering treatment pattern and core drugs of TCM prescriptions [30, 31]. Zhou et al. [23] designed a core drug discovery method based on effect degree. As a result, they found core drugs in consumptive lung disease prescription. Lu et al. [27] constructed a Chinese herbal medicine network by the National Health Insurance Research Database in Taiwan, where drugs are used for treating allergic rhinitis. They used social network analysis and association rules to explore the network and found most frequently used Xin-Yi-Qing-Fei decoction. Ma et al. [28] built a relation graph of drugs, syndromes, diseases, and therapies in TCM prescriptions and discovered 9 core drugs for treating gastric abscess by computing the degree, closeness centrality, and betweenness of the graph. Recently, Zhang et al. [22] proposed an artificial intelligence model to discover core drugs from literature by searching 1126 literature about treating chronic glomerulonephritis in TCM and designing a semantic analysis method to extract the meanings of drugs, construct drug network, and find three drug communities and 18 core drugs for curing various syndromes of chronic glomerulonephritis.

Above research studies can discover core drugs effectively, but artificial analysis and medical tests are only suitable for small-scale samples. Meanwhile, medical records need to preprocess manually to form structured data. Most of data mining approaches do not analyse the internal meanings of drugs in medical records. It is important that there are many literatures. In this paper, we combine word embedding and community detection to focus on literature analysis to extract the semantics of drugs in large-scale literature and identify core drugs for treating CPD.

## 3. The Learning Framework

In this paper, we design a learning framework CDDF for discovering core drugs for curing CPD with the purpose of importing the knowledges and semantics of Chinese drugs implied in large-scale literature. In CDDF, we analyse the drug semantics in literature by adopting Chinese word embedding model SSP2VEC [32], compute their semantic similarity to construct drug network, and identify core drugs in the drug network by community detection algorithm COPRA [33], which contains disease corpus construction, drug network generation, and core drug discovery stages, as presented in Figure 1. Two doctors independently evaluate the results of drug communities and core drugs to conduct quality assessment and give the analysis of experiment results according to the Pharmacopoeia of the People's Republic of China [34]. Each core drug is rated as true core drug, false core drug, or uncertain core drug. When there is any disagreement, it is resolved through discussion with the third doctor to obtain consensus.

### 3.1. Disease Corpus Construction

In the first stage, we collect large-scale literature about the treatment of CPD from CNKI and construct disease corpus *C* for training SSP2VEC. All sentences in literature are divided into Chinese words, and the unrelated information is removed (Algorithm 1).

 
*Step* 1. *Literature Acquisition.*
  According to the suggestions of TCM doctors, we choose two key Chinese word pairs (1) “伤寒 (cold pathogenic disease)” and “中医 (Chinese medicine)” and (2) “伤寒 (cold pathogenic disease)” and “中药 (Chinese native medicine)” to search relevant literature in CNKI. The full texts of all relevant literature are extracted, and drugs are included in these texts.
   *Step* 2. *Redundant Information Removal.*
   When we extract the contents of literature, there are some redundant information, such as messy code and punctuation, which has no implication in the original text. The characters whose Unicode belongs to the range between 0x4E00 and 0x9FA5 are Chinese characters; then, we retain them by regular expression and remove other information to obtain pure corpus.
   *Step* 3. *Font Conversion.*
   Chinese literature may contain traditional Chinese characters, and we convert them to simplified Chinese characters by the OpenCC toolkit (https://github.com/BYVoid/OpenCC) for uniformly processing.
   *Step* 4. *Word Segmentation.*
   Chinese sentences are comprised by connective words; then, we apply word segmentation algorithm [35] to divide Chinese sentences into independent words for extracting drug words.

### 3.2. Drug Network Generation

In the second stage, the sematic vectors of Chinese drugs are generated by SSP2VEC; then, the semantic similarity among drugs is computed to measure the similar degree of drug efficacy. Drug network *G* is built according to their semantic similarity. The drugs are considered as nodes, and if the similarity of two drugs is greater than similarity threshold *s*, then the edges are formed between the two drugs. The semantic vectors of Chinese drugs contain drug attributes (e.g., usage, efficacy, and taboo) and therapeutic relations between drugs and syndromes; then, the drug network can reflect drug attributes and treating syndromes in literature (Algorithm 2).

 *Step* 1. *Word Embedding.*
 Chinese drugs are recorded as Chinese words in literature. In the step, we adopt Chinese word embedding model SSP2VEC based on the stroke, structure, and pinyin to mine the meanings of Chinese drugs in literature [32]. Here, we briefly introduce word embedding and the theory of SSP2VEC. Word embedding models can capture word meanings according to the distributional hypothesis that similar semantic words tend to occur in similar contextual words, which illustrates that word semantics are contained in their contexts [36]. For example, there is a Chinese sentence “伤寒初感, 始于太阳, 故以发汗为先。 (the patients suffer from cold pathogenic disease, which starts from Tai-Yang syndrome, then the patients appear sweating symptom first).” The Chinese word “太阳 (Tai-Yang syndrome)” is chosen as the target word; then, we can gain its contextual words “伤寒 (cold pathogenic disease),” “初感(suffer from),” “始于 (start from),” “故以 (then),” “发汗 (sweating symptom),” and “为先 (first).” Although word embedding models cannot understand the accurate meaning of “太阳 (Tai-Yang syndrome),” they can know that the target word is related to its contextual words, which include relevant words such as “伤寒 (cold pathogenic disease)” and “发汗 (sweating symptom)” reflecting the disease and symptom of Tai-Yang syndrome. With the increase of training sentences, the methods can understand word semantics more and more accurately. Thus, we can forecast the target word according to its contexts or forecast the contexts according to the target word to learn their semantic representation. In order to intuitively understand semantic vectors, we visualize some Chinese drugs in the two-dimension coordinate system based on semantic vectors. As presented in Figure 2, we find that word embedding models can better differentiate different types of drugs and understand the semantics of these drugs, for example, they capture the drugs with similar efficacy, relieving superficies (麦冬 (*dwarf lilyturf tuber*), 玉竹 (*fragrant solomonseal rhizome*), and 沙参 (*coastal glehnia root*)), activating qi and digestive (陈皮 (*dried tangerine peel*) and 青皮 (*immature tangerine peel*)), and activating blood circulation (白芍 (*debark peony root*) and 赤芍 (*peony root*)). In large-scale literature, we can mine the meanings of Chinese drugs by word embedding models and represent them as low-dimension semantic vectors; then, the meanings of Chinese drugs are contained in the semantic vectors in a certain extent.
 Specially, Chinese words consist of characters that include inner attributes with rich semantics [30, 37]. There are many Chinese word embedding methods that have been proposed for mining the semantics of Chinese words with the character attribute [38] and the inner-character attributes of Chinese words, such as radical [39], component [40], and stroke *n*-gram [41]. For example, there is a Chinese character “怹 (the honorific of he),” in which its radical is “心 (heart),” its components are “亻 (people),” “也 (also),” and “心 (heart),” and its stroke *n*-grams include “亻 (people),” “也 (also),” “他 (he),” and “心 (heart).” Among these parts, stroke *n*-gram “他 (he)” is the most related to the entire character because “怹” is the honorific of “他.” It can be seen that stroke *n*-gram feature includes radical and component attributes and can understand some meanings of “怹 (the honorific of he).” Meanwhile, “怹 (the honorific of he)” is a character of up-down structure and “他 (he)” is on the top of “心 (heart).” This up-down structure can demonstrate that he is on my heart (i.e., you are in my heart.) to reflect the implication of honorific. Besides stroke and structure features, the pronunciation of Chinese characters (pinyin) also can support the model to capture the semantics of onomatopoeia and differentiate the Chinese characters that own the same stroke *n*-gram and structure features [32]. For example, the pinyin of “汪汪 (bark)” is “wāng wāng.” When we hear the pronunciation, we can understand its sense is the sound of the dog. Thus, we adopt SSP2VEC in CDDF to mine the meanings of Chinese words according to the inner-character attributes (stroke, structure, and pinyin).
 The framework of SSP2VEC is presented in Figure 3. For the Chinese sentence “伤寒初感，始于太阳，故以发汗为先。 (the patients suffer from cold pathogenic disease, which starts from Tai-Yang syndrome, then the patients appear sweating symptom first.),” the target word is “太阳 (Tai-Yang syndrome),” and its contexts are “伤寒 (cold pathogenic disease),” “初感 (suffer from),” “始于 (start from),” “故以 (then),” “发汗 (sweating symptom),” and “为先 (first).” SSP2VEC is made up of five parts as follows.
  (1) Input part: the first part is to accept target word *w*_*t*_, for example, “太阳 (Tai-Yang syndrome).”
  (2) Feature extraction part: the second part is utilized to divide word *w*_*t*_ into a single character, for example, “太” and “阳,” and extract the inner-character attributes of each character (e.g., stroke, structure, and pinyin).
  (3) Feature encoding part: the third part is designed to encode the stroke, structure, and pinyin attributes according to the codes defined in [32]. For example, for the Chinese word “太阳 (Tai-Yang syndrome),” the stroke, structure, and pinyin codes of character “太” are “1344,” “96,” and “taiD,” respectively. The stroke, structure, and pinyin codes of character “阳” are “522511,” “66,” and “yangB,” respectively.
  (4) Feature substring generation part: the part is to assemble the inner-character attributes by generating the feature substring through moving a slide window with different lengths. For example, the feature substring of “太阳 (Tai-Yang syndrome)” can be generated by (1) forming the whole code sequence of this word in the order of stroke, structure, and pinyin as “134496taiD25241166yangB,” (2) setting the length of slide window *n* = 1 and moving the window on the whole sequence; then, we can get feature substrings as “1,” “3,” …, “g” and “B,” and (3) increasing the length of slide window and moving. We can obtain feature substrings as “13,” “34,”,…, “ng” and “gB” when *n* = 2. With the increase of window length (from one to the length of the entire sequence), we can get more feature substrings. For example, when *n* = 3, we can obtain feature substrings as “134,” “344,” …, “ang” and “ngB.” The feature substring can include radical, component, and stroke *n*-gram with structure and pinyin features. For example, feature substring “52” denotes the radical of “阳.”
  (5) Output part: output part is defined as *softmax* function [42] to compute the likelihood that the contexts of word *w*_*t*_ are forecast according to all feature substrings of word *w*_*t*_, which is optimized according to standard gradient methods [41].
SSP2VEC reads Chinese words on corpus according to the operation mode shown in Figure 4. Specifically, it reads target word *w*_*t*_ and *c* words before and after word *w*_*t*_ as its contexts. For example, SSP2VEC reads the words in the green ellipse as one record where the Chinese word in the red box as target word *w*_*t*_ and extracts the Chinese words in blue boxes as contextual words *C*_*t*_  of word *w*_*t*_ (*c* = 2). SSP2VEC traverses the whole corpus and analyses the semantics of different target words. When the training process is finished, we employ the semantic vectors of contexts as output results; then, we can gain semantic vectors *U* = {*u*_1_,…, *u*_*t*_,…, *u*_*N*′_} of Chinese words on corpus, where *u*_*t*_ is the semantic vector of word *w*_*t*_ and *N*′ denotes the number of nonrepeating words.
 *Step* 2. *Drug Extraction.*
 All Chinese words in corpus *C* are used to train SSP2VEC for learning the semantics of drugs because the contexts of words are necessary; then, we obtain semantic vectors; however, words include drugs, symptoms, syndromes, and other elements. Thus, we extract semantic vector set *U*_*H*_ of drugs where *H* is the drugs in collected literature [43]. The regulate drug name in the book the Pharmacopoeia of the People's Republic of China [34] is used to construct standard drug thesaurus *D*. If drugs are in corpus *C* and standard drug thesaurus *D* at the same time, then the drugs and their semantic vectors are extracted.
 *Step* 3. *Semantic Similarity Calculation.*
According to the meanings of drugs in literature, their semantic similarity can reflect the similar degree of efficacy, which illustrates that they can treat similar syndromes and diseases. If the semantic similarity among drugs is higher than a given similarity threshold *s*, then we can consider that they have similar efficacy and can cure similar diseases and syndromes. Cosine similarity is a good measurement to evaluate similarity [44]; then, the semantic similarity of drugs is calculated according to cosine similarity, which is defined as
  (1) $$\begin{array}{c} \text{similarity}\left(w_{i},w_{j}\right)=\frac{u_{i}\cdot u_{j}}{\left|u_{i}\right|\left|u_{j}\right|}. \end{array}$$
 *Step* 4. *Drug Network Generation.*
 The drug network is built by drugs with semantic similarity. We consider the drugs as nodes, and if their similarity is greater than similarity threshold *s*, then the edges form between them.

### 3.3. Core Drug Discovery

In the stage, core drug set *D*^core^ = {*D*_1_^core^,…, *D*_*i*_^core^,…, *D*_*K*_^core^} is discovered in drug community *O* = {*O*^1^,…, *O*^*i*^,…, *O*^*K*^} in the drug network, in which *K* denotes the number of drug communities (Algorithm 3).

   *Step* 1. *Drug Community Discovery.*
  Drugs in drug communities have similar efficacy to treat one class syndrome of CPD. Community structures are the partition of a network into node groups owing dense internal links and sparse interconnections [33]. Community detection methods can discover node division and classification with similar attributes, which is beneficial for effectively analysing networks. For instance, discovering groups in hobby networks might detect the interest communities, and discovering groups in drug networks might detect the drugs having similar efficacy. COPRA is an effective community detection algorithm [33]. When COPRA stops, if nodes have the same label, then they are assigned to the same community [33]. The corresponding concepts between COPRA and core drug discovery are shown in Table 1. Thus, we introduce COPRA in CDDF for detecting drug communities and core drugs in the drug network.
  Given an example in Figure 5 to explain the process of COPRA, the node representing Chinese drug 麦冬 (*dwarf lilyturf tuber*) is selected for updating its labels at first. The neighbouring nodes launch their labels owning belonging coefficients to this node, whose belonging coefficients are assumed to 1; then, node 麦冬 (*dwarf lilyturf tuber*) receives labels: (yellow, 1), (yellow, 1), (yellow, 1), (pink, 1), (pink, 1), and (green, 1). We gain this node with labels (yellow, 3/6), (pink, 2/6), and (green, 1/6) by normalizing their belonging coefficients. If the belonging coefficient is less than 1/*r* (threshold *r* equals to 2), then the pink and green labels are removed. As a result, we update the label of node 麦冬 (*dwarf lilyturf tuber*) to the yellow label; then, this node is allocated to the yellow group, where drugs have similar efficacy (e.g., relieving superficies). The above process conducts iteratively until the labels of nodes remain unchanged. Finally, the nodes are assigned to the communities characterized by their labels. When the method is finished, three communities are discovered. As shown in Figure 6, the procedures of COPRA contain six steps initialization, node choice, label launch, label acceptation, termination judgement, and postprocessing [33].
   *Step* 2. *Core Drug Discovery.*
   In each community, if the drug nodes have large degree, we consider that they are pivotal. Meanwhile, there are 8–10 core drugs for treating one syndrome of CPD in TCM [21]. Thus, we choose ten drugs owning the top-10 degree in every community as core drugs, which have the efficacy representing by corresponding community for treat one class syndrome of CPD.

## 4. Experiential Results and Discussion

In the section, the experiments are conducted on the disease corpus. We adopt the open database CNKI to collect relevant literature so that there are no ethical issues. After searching in CNKI by the key word pairs, we collect 4681 literature about the TCM treatment of CPD and process them according to stage 1; then, disease corpus is built with 50 million tokens. All literature are relevant to the treatment of CPD in TCM, so we can axcept that semantic analysis can better understand the semantics of Chinese drugs and obtain good semantic vectors. Then, we apply CDDF in the corpus to discover core drugs for treating CPD comparing with CSG + COPRA, in which continuous skip-gram (CSG) model is a state-of-the-art word embedding model [42] but does not consider the inner-character attributes (stroke, structure, and pinyin).

The results of drug communities and core drugs are shown in Figure 7. As shown in Figure 7(a), the drug network owning 316 nodes and 251 edges is established by CDDF, and CDDF discovers 12 major drug communities. As shown in Figure 7(b), the drug network owning 316 nodes and 281 edges is established by the comparing method, and it detects 10 drug communities. There are some isolated nodes in drug networks because some Chinese drugs may have no relationship with other drugs according to the collected literature or their similarity is less than the similarity threshold. Thus, we present and colour the communities with more than three nodes and then resize nodes in the descending order of degree. Finally, we choose top-10 drugs in each community as core drugs for treating one CPD syndrome.

According to *the Pharmacopoeia of the People's Republic of China* [34], which records the efficacy and indication (therapeutic syndrome and symptom) of drugs, after discussing with three Chinese medicine doctors, they consider that the core drugs discovered by the proposed framework are more realistic and effective than the comparing method for treating CPD. First, two Chinese medicine doctors analyse the experiential results independently. If they have different comments, then they discuss with the third doctors and obtain consensus. As mentioned above, the drugs in the same drug community denote that they own similar function and efficacy and can treat similar symptoms of one syndrome of CPD. For explaining the advantage of the proposed model, we show the details of some drug communities in Figures 8 and 9 (in each community, for the drugs owning top-10 degree, the drugs in the red circle denote the core drugs for curing one syndrome of CPD, the drugs in the blue circle means that they can compose a classic prescription with supporting drugs for treating one syndrome of CPD, and the drugs in the green circle are the supporting drugs for treating CPD). We can find that some drugs belong to two communities (e.g., *liquorice root* (甘草) shown in the communities of Figures 8(a) and 8(b) and *prepared common monkshood branched root* (附子) shown in the communities of Figures 8(a) and 8(c)) since they are important drugs or play reconcile function in the two communities. The details of these communities are shown in Tables 2 and 3 where the drugs labelled with the bold font are correctly identified as related drugs.

According to the analysis of TCM doctors with *the Pharmacopoeia of the People's Republic of China* [34] as standard, as shown in Figure 8(a), all drugs in the red community are the core drugs for Tai-Yang syndrome of CPD. They have the efficacy of relieving superficies syndrome with pungent and warm natured drugs (辛温解表). Five Chinese drugs *liquorice root* (甘草), *fresh ginger* (生姜), *paeonia lactiflora pall* (芍药), *cassia twig* (桂枝), and *Chinese date* (大枣) in the red community can compose Gui-Zhi decoction which is the primary prescription for treating Tai-Yang syndrome of CPD. As shown in Figure 8(b), the seven drugs in red circles in the green community are the core drugs for treating Tai-Yin syndrome of CPD. They have the efficacy of benefiting vital energy and invigorating spleen (益气健脾). Four Chinese drugs *liquorice root* (甘草), *largehead atractylodes rhizome* (白术), *tangshen* (党参), and *Indian bread* (茯苓) can form the main prescription for treating Tai-Yin syndrome of CPD, which is called as Si-Jun-Zi decoction. We can add other drugs in red circles except the four drugs in Si-Jun-Zi decoction to enhance the efficacy of invigorating spleen. The *liquorice root* (甘草) belongs to the red and green communities simultaneously because it is a harmonizing drug in the two classic prescriptions. As shown in Figure 8(c), all drugs in the light green community are the core drugs for treating Shao-Yin syndrome of CPD, which have the efficacy of strengthening body resistance for relieving superficies syndrome (扶正解表). Three Chinese drugs *ephedra* (麻黄), *prepared common monkshood branched root* (附子), and *manchurian wildginger* (细辛) can compose Ma-Huang-Fu-Zi-Xi-Xin decoction which is the important prescription for treating Shao-Yin syndrome of CPD and is always used in the treatment of influenza. The *bitter apricot seed* (杏仁) and *platycodon root* (桔梗) can regulate the function of lungs and enhance the effectiveness of Ma-Huang-Fu-Zi-Xi-Xin decoction. The *prepared common monkshood branched root* (附子) belongs to the green and light green communities at the same time because it owns two efficacies with equal importance. As shown in Figure 8(d), the six drugs in red circles in the blue community own the efficacy of activating blood circulation. The *safflower* (红花), *debark peony root* (白芍), *sichuan lovage rhizome* (川芎), *peach seed* (桃仁), and *Chinese angelica* (当归) are the five drugs of the classical prescription Tao-Hong-Si-Wu decoction for activating blood circulation. However, there lacks *prepared rehmannia root* (熟地黄), which has the efficacy of invigorating the kidney mainly; thus, it is assigned to that community representing the efficacy of invigorating the kidney. As shown in Figure 8(e), the seven drugs in green circles in the dark purple community are the representative drugs with the efficacy of activating qi and digestive (行气消食). However, they are not the core drugs for treating CPD. According to the analysis of TCM doctors, these drugs can assist the core drugs to reduce the secondary symptoms of patients. As shown in Figure 8(f), the eight drugs in green circles in the light purple community own the efficacy of expelling superficial evils and clearing away the heat-evil (清热解毒). However, they are also not the core drugs for treating CPD. They are the representative drugs with the efficacy of expelling superficial evils and clearing away the heat-evil to enhance the efficacy of core drugs.

Comparing with the proposed framework, the CSG + COPRA method only can detect the drug communities where drugs own the same efficacy and important drugs with corresponding efficacy; however, they are not for treating CPD. As shown in Figure 9(a), five drugs in green circles in the blue community have the efficacy of activating blood circulation. However, they are not the core drugs for treating CPD. As shown in Figure 9(b), only *prepared rehmannia root* (熟地黄) is discovered correctly as the core drug for treating CPD. The six drugs in green circles in the pink community have the efficacy of invigorating the kidney and can enhance the physique of humans. However, they are not the core drugs for treating CPD. As shown in Figure 9(c), the nine drugs in green circles in the dark purple community have the efficacy of activating qi and digestive. They can enhance the physique of human support core drugs to cure CPD. As shown in Figure 9(d), only the *glabrous greenbrier rhizome* (土茯苓) is found correctly as the core drug. The five drugs in green circles in the light purple community own the efficacy of clearing away the heat-evil and expelling superficial evils.

In summary, the proposed framework finds most core drugs with high accuracy for treating CPD and four classical prescriptions to deal with the different stages of CPD from large-scale literature, which shows that SSP2VEC considers that the inner-character attributes (stroke, structure, and pinyin) can better understand the semantics of drugs in literature than CSG. Meanwhile, it also discovers some drugs to support the core drugs for treating CPD. CDDF can assist doctors by rapidly analysing large-scale literature, but the medication usage should be made by doctors. In contrast, CSG + COPRA gets poorer accuracy than CDDF since it only finds important drugs with the same efficacy and cannot find the core drugs for treating CPD. CSG cannot understand more semantics of Chinese drugs than SSP2VEC. Of course, SSP2VEC also cannot understand the complete meanings of drugs in literature since the corpus scale is limit. In general, we can find that CDDF discovers most correct core drugs for curing different CPD syndromes.

In order to further research the drug network built by the proposed framework, we compute its community size, closeness centrality, and degree distributions to analyse the patterns of core drugs, whose results are shown in Figure 10 and Table 4.

1. Community size distribution reflects the node number in each community, and we can find main drug communities according to this distribution. As shown in Figure 10(a), there are 12 communities with more than two nodes (e.g., 23, 3, 11, 4, 18, 10, 8, 10, 12, 4, 4, and 3); especially, six communities own more than 10 nodes (e.g., 23, 11, 18, 10, 10, and 12). In these communities, core drugs and four classical prescriptions are identified for treating different syndromes of CPD. Other communities only have one or two nodes, which may be because literature contain multiple syndromes and symptoms of patients, and the drugs in small drug communities are adopted to cure the patients' secondary symptoms. Meanwhile, core drugs are discovered in major communities, which demonstrates that core drugs are frequently used with other drugs for treating CPD. As a result, core drugs are detected from major drug communities to cure the syndromes of CPD in TCM.
2. Closeness centrality distribution reflects the node number owning different closeness, which is the measurement of node centrality in the network. In the red community, the closeness centrality of core drugs is 0.24, 0.20, 0.22, 0.21, 0.17, 0.19, 0.19, 0.15, and 0.19, respectively, which focuses on the range of [0.15, 0.24], as shown in Table 4. In other communities, the closeness centrality of core drugs focuses on the range of [0.16, 0.27], [0.13, 0.18], [0.15, 0.25], [0.19, 0.28], and [0.12, 0.18], respectively. Thus, we consider that the closeness centrality of core drugs for treating CPD is in the range of [0.10, 0.30]. However, closeness centrality is an evaluation metric to identify core nodes in networks; then, the nodes with large centrality may be considered as core nodes in networks. According to the experimental results, core drugs have small centrality (i.e., [0.10, 0.30]); in other words, core drugs for treating CPD are not corresponding to central core nodes in networks but to nodes with small closeness centrality, as shown in Figure 10(b).
3. Degree distribution reflects the node number owning different degrees, which is the measurement of node importance in networks. In the red community, the degree of core drugs is 8, 6, 4, 4, 3, 2, 2, 2, and 1, respectively, which is less than 8, as shown in Table 4. In other communities, the degree of core drugs is less than 8, 4, 8, 13, and 7, respectively. Thus, we consider that the degree of core drugs for treating CPD is less than 13, as shown in Figure 10(c). Under this range, the larger degree is, the more important node is; then, core drugs can be regarded as the important nodes in networks, which is consistent with the definition that degree can reflect node importance in networks. As presented in Figure 10(c), the degree of important core drugs focuses in the range of [4.0, 10.0]. Thus, we can think that core drugs have large degree and small closeness centrality, that is, core drugs are important nodes but not central nodes in networks.

## 5. Conclusions

In this paper, we explore core drug discovery for treating CPD in TCM from large-scale literature. A learning CDDF containing three steps (disease corpus construction, drug network generation, and core drug discovery) is proposed based on word embedding and community detection. Chinese word embedding model SSP2VEC is used for mining the meanings of Chinese drugs in literature; then, the drug network is built by their semantic similarity. Community detection algorithm COPRA is adopted to find drug communities, and the key nodes with large degree in every drug community are considered as core drugs. The proposed framework can reveal better and effective drug communities and core drugs. Thus, CDDF can be used to identify core drugs for treating specific diseases and assisting the decision-making of doctors.

However, we can find that some drugs are discovered in the drug network, which are not core drugs. Improving the proposed framework or designing new methods [45, 46] with domain knowledge to detect more accurate drug communities and core drugs is an important future work. The data source of literature and the number of words in literature have an influence on the results of semantic analysis, so selecting authoritative literature and enlarging corpus scale can increase the accuracy. In addition, selecting the literature of certain TCM doctor can analyse the treatment experience of this doctor, which is also an important research work in the future.

## Figures and Tables

**Figure 1:** The process of CDDF.

**Figure 2:** An example of semantic vectors.

**Figure 3:** The framework of SSP2VEC.

**Figure 4:** The operation mode of SSP2VEC.

**Figure 5:** An example of the updating of node labels.

**Figure 6:** COPRA's process.

**Figure 7:** The drug communities found by different models. (a) CDDF (SSP2VEC + COPRA). (b) The comparing method (CSG + COPRA).

**Figure 8:** The details of partial communities found by the proposed framework.

**Figure 9:** The details of partial communities found by the comparing algorithm.

**Figure 10:** Network analysis results. (a) Community size distribution. (b) Closeness centrality distribution. (c) Degree distribution.

**Algorithm 1:** Stage 1 disease corpus construction.

**Algorithm 2:** Stage 2 drug network generation.

**Algorithm 3:** Stage 3 core drug discovery.

**Table 1:** Corresponding relations.

Community detection	Core drug discovery
Node	Drug
Edge	The similar relation among drugs
Label	Drug efficacy
Communities	Drug groups for curing similar syndromes
Nodes with large degree in every community	Core drugs for curing one class syndromes

**Table 2:** Top-10 drugs in partial drug communities found by the proposed framework.

Community	Efficacy	Drug (English)	Drug (Chinese)
Red	Relieving superficies syndrome with pungent and warm natured drugs (辛温解表)	**Liquorice root**	**甘草**
		**Fresh ginger**	**生姜**
		**Paeonia lactiflora pall**	**芍药**
		**Cassia twig**	**桂枝**
		**Dried ginger**	**干姜**
		**Chinese date**	**大枣**
		**Pinellia tuber**	**半夏**
		**Prepared common monkshood branched root**	**附子**
		**Ginseng**	**人参**

Dark green	Benefitting vital energy and invigorating spleen (益气健脾)	**Liquorice root**	**甘草**
		**Largehead atractylodes rhizome**	**白术**
		**Tangshen**	**党参**
		**Oriental waterplantain rhizome**	**泽泻**
		Common yam rhizome	山药
		**Indian bread**	**茯苓**
		Gordon euryale seed	芡实
		**Milkvetch root**	**黄芪**
		**Zhuling**	**猪苓**
		Cherokee rose fruit	金樱子

Light green	Strengthening body resistance for relieving superficies syndrome (扶正解表)	**Ephedra**	**麻黄**
		**Manchurian wildginger**	**细辛**
		**Prepared common monkshood branched root**	**附子**
		**Bitter apricot seed**	**杏仁**
		**Platycodon root**	**桔梗**

Blue	Activating blood circulation (活血)	**Safflower**	**红花**
		Danshen root	丹参
		**Debark peony root**	**白芍**
		Peony root	赤芍
		**Sichuan lovage rhizome**	**川芎**
		**Peach seed**	**桃仁**
		**Chinese angelica**	**当归**
		Suberect spatholobus stem	鸡血藤
		Hirsute shiny bugleweed drug	泽兰
		**Rhubarb root and rhizome**	**大黄**

Dark purple	Activating qi and digestive (行气消食)	**Dried tangerine peel**	**陈皮**
		**Common aucklandia root**	**木香**
		**Immature tangerine peel**	**青皮**
		**Nutgrass galingale rhizome**	**香附**
		Yanhusuo	延胡索
		**Villous amomum fruit**	**砂仁**
		**Orange fruit**	**枳壳**
		Finger citron	佛手
		Turmeric root tuber	郁金
		**Medicated leaven**	**神曲**

Light purple	Expelling superficial evils and clearing away the heat-evil (清热解毒)	**Isatis root**	**板蓝根**
		**Dandelion**	**蒲公英**
		**Honeysuckle bud and flower**	**金银花**
		**Heartleaf houttuynia drug**	**鱼腥草**
		**Weeping forsythia capsule**	**连翘**
		**Wild chrysanthemum flower**	**野菊花**
		Fern rhizome	贯众
		**Tokyo violet drug**	**紫花地丁**
		**Atrina glass**	**败酱草**
		Great burdock achene	牛蒡子

**Table 3:** Top-10 drugs in the partial drug community found by the comparing method.

Community	Efficacy	Drug (English)	Drug (Chinese)
Blue	Activating blood circulation (活血)	India madder root	茜草
		**Myrrh**	**没药**
		Cattail pollen	蒲黄
		**Frankincense**	**乳香**
		**Pangolin scales**	**穿山甲**
		Hirsute shiny bugleweed drug	泽兰
		**Sappan wood**	**苏木**
		**Suberect spatholobus stem**	**鸡血藤**
		Kadsura pepper stem	海风藤
		Garden burnet root	地榆

Pink	Invigorating the kidney (补肾)	**Dodder seed**	**菟丝子**
		**Chinese taxillus drug**	**桑寄生**
		**Eucommia bark**	**杜仲**
		Cherokee rose fruit	金樱子
		Solomonseal rhizome	黄精
		**Glossy privet fruit**	**女贞子**
		**Degelatined deer-horn**	**鹿角霜**
		**Deer-horn glue**	**鹿角胶**
		**Prepared rehmannia root**	**熟地黄**
		**Himalayan teasel root**	**续断**

Dark purple	Activating qi flowing and digestive (行气消食)	**Medicated leaven**	**神曲**
		**Germinated barley**	**麦芽**
		**Finger citron**	**佛手**
		**Inner membrane of chicken gizzard**	**鸡内金**
		**Hawthorn fruit**	**山楂**
		**Common aucklandia root**	**木香**
		**Villous amomum fruit**	**砂仁**
		**Immature tangerine peel**	**青皮**
		Millet sprout	谷芽
		**Radish seed**	**莱菔子**

Light purple	Expelling superficial evils and clearing away the heat-evil (清热解毒)	**Atrina glass**	**败酱草**
		**Dandelion**	**蒲公英**
		**Arnebia root**	**紫草**
		**Heartleaf houttuynia drug**	**鱼腥草**
		Giant knotweed rhizome	虎杖
		**Glabrous greenbrier rhizome**	**土茯苓**
		**Isatis root**	**板蓝根**
		Fern rhizome	贯众

**Table 4:** The degree and closeness centrality of top-10 drugs in partial communities.

Community	Drug (English)	Drug (Chinese)	Closeness centrality	Degree
Red	**Liquorice root**	**甘草**	**0.24**	**8**
	**Fresh ginger**	**生姜**	**0.20**	**6**
	**Paeonia lactiflora pall**	**芍药**	**0.22**	**4**
	**Cassia twig**	**桂枝**	**0.21**	**4**
	**Dried ginger**	**干姜**	**0.17**	**3**
	**Chinese date**	**大枣**	**0.19**	**2**
	**Pinellia tuber**	**半夏**	**0.19**	**2**
	**Prepared common monkshood branched root**	**附子**	**0.15**	**2**
	**Ginseng**	**人参**	**0.19**	**1**

Dark green	**Liquorice root**	**甘草**	**0.24**	**8**
	**Largehead atractylodes rhizome**	**白术**	**0.27**	**8**
	**Tangshen**	**党参**	**0.25**	**5**
	**Oriental waterplantain rhizome**	**泽泻**	**0.22**	**4**
	Common yam rhizome	山药	0.23	4
	**Indian bread**	**茯苓**	**0.21**	**2**
	Gordon euryale seed	芡实	0.19	2
	**Milkvetch root**	**黄芪**	**0.21**	**1**
	**Zhuling**	**猪苓**	**0.18**	**1**
	Cherokee rose fruit	金樱子	0.16	1

Light green	**Ephedra**	**麻黄**	**0.18**	**4**
	**Manchurian wildginger**	**细辛**	**0.15**	**3**
	**Prepared common monkshood branched root**	**附子**	**0.15**	**2**
	**Bitter apricot seed**	**杏仁**	**0.15**	**3**
	**Platycodon root**	**桔梗**	**0.13**	**3**

Blue	**Safflower**	**红花**	**0.19**	**8**
	Danshen root	丹参	0.22	8
	**Debark peony root**	**白芍**	**0.25**	**8**
	Peony root	赤芍	0.21	6
	**Sichuan lovage rhizome**	**川芎**	**0.21**	**5**
	**Peach seed**	**桃仁**	**0.18**	**4**
	**Chinese angelica**	**当归**	**0.20**	**4**
	Suberect spatholobus stem	鸡血藤	0.18	3
	Hirsute shiny bugleweed drug	泽兰	0.16	3
	**Rhubarb root and rhizome**	**大黄**	**0.15**	**2**

Dark purple	**Dried tangerine peel**	**陈皮**	**0.28**	**13**
	**Common aucklandia root**	**木香**	**0.24**	**10**
	**Immature tangerine peel**	**青皮**	**0.24**	**9**
	**Nutgrass galingale rhizome**	**香附**	**0.24**	**8**
	Yanhusuo	延胡索	0.20	7
	**Villous amomum fruit**	**砂仁**	**0.23**	**7**
	**Orange fruit**	**枳壳**	**0.23**	**6**
	Finger citron	佛手	0.19	6
	Turmeric root tuber	郁金	0.23	6
	**Medicated leaven**	**神曲**	**0.22**	**5**

Light purple	**Isatis root**	**板蓝根**	**0.16**	**7**
	**Dandelion**	**蒲公英**	**0.14**	**7**
	**Honeysuckle bud and flower**	**金银花**	**0.15**	**6**
	**Heartleaf houttuynia drug**	**鱼腥草**	**0.14**	**5**
	**Weeping forsythia capsule**	**连翘**	**0.18**	**4**
	**Wild chrysanthemum flower**	**野菊花**	**0.14**	**4**
	Fern rhizome	贯众	0.13	3
	**Tokyo violet drug**	**紫花地丁**	**0.12**	**3**
	**Atrina glass**	**败酱草**	**0.12**	**3**
	Great burdock achene	牛蒡子	0.13	2

The drugs labeled with bold values are correctly identified related drugs.

## Data Availability

The text data used to support the findings of this study have been deposited in https://github.com/yunzhangwww/CPD-literature-corpus.

## References

[1] Wang Q. G., Li J. T., He X. H. (2016). *The Selected Readings of Treatise on Cold Pathogenic Disease*.

[2] Luo H.-h., Zhang F.-x., Wu W., Wang X.-h. (2016). Haoqin Qingdan Decoction (蒿芩清胆汤) and ribavirin therapy downregulate CD14 and toll-like receptor 4 in febrile disease with dampness-heat syndrome in a mouse model. *Chinese Journal of Integrative Medicine*.

[3] Zhao L. C. (2011). Discussion on the internal and external disease causes in syndrome differentiation of exogenous fever. *Journal of Traditional Chinese Medicine*.

[4] Tansey T. (2020). The pandemic bookshelf grows. *Nature*.

[5] Li Q., Liu Y. T., He Z. Y. (2014). Ancient literature research on exogenous fever of traditional Chinese medicine based on bibliometrics content analysis. *Journal of Guangzhou University of Traditional Chinese Medicine*.

[6] Du M. B. (2019). Discussion on drug dosage in treatise on febrile diseases. *Zhongguo Zhongyao Zazhi*.

[7] Li Y., Xue Y. X. (2015). Preliminary study on the principles and methods of professor Xue- Bo-Shou’s treating exogenous febrile disease. *China Journal of Traditional Chinese Medicine and Pharmacy*.

[8] Wu L., Chen Y., Ma Y. (2020). Clinical practice guideline on treating influenza in adult patients with Chinese patent medicines. *Pharmacological Research*.

[9] Li X. Y., Lundborg C. S., Ding B. H. (2018). Clinical outcomes of influenza-like illness treated with Chinese herbal medicine: an observational study. *Journal of Traditional Chinese Medicine*.

[10] Ginsberg J., Mohebbi M. H., Patel R. S., Brammer L., Smolinski M. S., Brilliant L. (2009). Detecting influenza epidemics using search engine query data. *Nature*.

[11] Song X., Xiao J., Deng J., Kang Q., Zhang Y., Xu J. (2016). Time series analysis of influenza incidence in Chinese provinces from 2004 to 2011. *Medicine*.

[12] Wang R. B., Li X. W., Chen X. R. (2015). Analysis on feature of TCM syndrome in 975 cases of influenza patients. *Journal of Traditional Chinese Medicine*.

[13] Yue D. H., Bi Y., Song Y. (2015). Research on TCM treatment of influenza. *China Journal of Traditional Chinese Medicine and Pharmacy*.

[14] Jia C. H. (2020). Questioning etiology and pathogenesis theory of traditional Chinese medicine: taking Tai-yang wind-stroke pattern and Gui-Zhi decoction in Shanghan Lun as an example. *Journal of Beijing University of Traditional Chinese Medicine*.

[15] Yu X., Cui Z., Zhou Z., Shan T., Li D., Cui N. (2014). Si-Jun-Zi decoction treatment promotes the restoration of intestinal function after obstruction by regulating intestinal homeostasis. *Evid Based Complement Alternat Med*.

[16] Li J., Lian J. W., Zhou Y. X. (2012). *Formula of Traditional Chinese Medicine*.

[17] Xu H. Y., Zhang Y. Q., Liu Z. M. (2019). ETCM: an encyclopaedia of traditional Chinese medicine. *Nucleic Acids Research*.

[18] Zhu J., Liu Y., Zhang Y. (2019). IHPreten: a novel supervised learning framework with attribute regularization for prediction of incompatible herb pair in traditional Chinese medicine. *Neurocomputing*.

[19] Bai Y. J. (2014). *Design, Synthesis, and Biological Characterization of Drug Molecules Based on “Jun-Chen-Zuo-Shi” Strategy*.

[20] Wu L., Wang Y., Li Z., Zhang B., Cheng Y., Fan X. (2014). Identifying roles of “Jun-Chen-Zuo-Shi” component herbs of QiShenYiQi formula in treating acute myocardial ischemia by network pharmacology. *Chinese Medicine*.

[21] Zhang Y., Liu Y., Jin R., Li Q., Jin R., Wen C. (2020). LILPA: a label importance based label propagation algorithm for community detection with application to core drug discovery. *Neurocomputing*.

[22] Zhang Y., Liu Y. G., Zhu J. J., Zhai S., Jin R., Wen C. (2020). A semantic analysis and community detection based artificial intelligence model for core herb discovery from the literature: taking chronic glomerulonephritis treatment as a case study. *Computational and Mathematical Methods in Medicine*.

[23] Zhou W., Wang F., Wang C. J., Xie J. Y. (2013). Mining core herbs and their combination rules using effect degree. *Journal of Frontiers of Computer Science & Technology*.

[24] Lin Z. Y., Lin J. R., Wan W. R. (2018). Compatibility of monarch, minister, assistant and guide in acupuncture prescription. *Journal of Traditional Chinese Medicine*.

[25] Lin Y. H., Huang M. D. (2019). Importance of monarch-minister-assistant-envoy in the prescription of Chinese medicine. *Clinical Journal of Chinese Medicine*.

[26] Yan S., Zhang R., Zhou X., Li P., He L., Liu B. (2013). Exploring effective core drug patterns in primary insomnia treatment with Chinese herbal medicine: study protocol for a randomized controlled trial. *Trials*.

[27] Lu Y. C., Yang C. W., Lin Y. H. (2020). Identifying the Chinese herbal medicine network and core formula for allergic rhinitis on a real-world database. *Evidence-based Complementary and Alternative Medicine*.

[28] Ma Y., Zhang D., Wulamu A., Xie Y., Zang H., Zhang J. (2014). The core drugs analysis based on social network analysis about traditional Chinese medicine records semantic relation. *Procedia Computer Science*.

[29] Huang Z., Juarez J. M., Li X. (2017). Data mining for biomedicine and healthcare. *Journal of Healthcare Engineering*.

[30] He L., Zhou Z. Y., Niu F. S. (2020). Research on standard compliance test algorithm based on electronic medical records of traditional Chinese medicine outpatients. *Journal of Healthcare Engineering*.

[31] Choi M. J., Choi B. T., Shin H. K., Shin B. C., Han Y. K., Baek J. U. (2015). Establishment of a comprehensive list of candidate antiaging medicinal herb used in Korean medicine by text mining of the classical Korean medical literature, Dongeuibogam, and preliminary evaluation of the antiaging effects of these herbs. *Evidence-Based Complementary and Alternative Medicine*.

[32] Zhang Y., Liu Y. G., Zhu J. J. Learning Chinese word embeddings from stroke, structure and pinyin of characters.

[33] Gregory S. (2010). Finding overlapping communities in networks by label propagation. *New Journal of Physics*.

[34] State Pharmacopoeia Commission of the PRC (2010). *Pharmacopoeia Commission of the Ministry of Health of the People’s Republic of China, the Pharmacopoeia Of the People’s Republic of China*.

[35] Gan L., Zhang Y. (2020). Investigating self-attention network for Chinese word segmentation. *IEEE/ACM Trans. Audio Speech Lang. Process*.

[36] Harris Z. S. (1954). Distributional structure. *Word*.

[37] Meng Y. X., Wu W., Wang F. Glyce: glyph-vectors for Chinese character representations.

[38] Chen X. X., Lei X., Liu Z. Y., Sun M. S., Luan H. B. Joint learning of character and word embeddings.

[39] Sun Y. M., Lin L., Yang N., Ji Z. Z., Wang X. L. Radical-enhanced Chinese character embedding.

[40] Yu J. X., Jian X., Xin H., Song Y. Q. Joint embeddings of Chinese words, characters, and fine-grained sub-character components.

[41] Cao S. S., Lu W., Zhou J., Li X. L. Cw2vec: learning Chinese word embeddings with stroke n-gram information.

[42] Mikolov T., Chen K., Corrado G., Dean J. (2013). Efficient Estimation of Word Representations in Vector Space. https://arxiv.org/abs/1301.3781.

[43] Liang J., Xian X., He X. (2017). A novel approach towards medical entity recognition in Chinese clinical text. *Journal of Healthcare Engineering*.

[44] Abdel-Basset M., Mohamed M., Elhoseny M., Son L. H., Chiclana F., Zaied A. E.-N. H. (2019). Cosine similarity measures of bipolar neutrosophic set for diagnosis of bipolar disorder diseases. *Artificial Intelligence in Medicine*.

[45] Sun W., Cai Z., Li Y., Liu F., Fang S., Wang C. (2018). Data processing and text mining technologies on electronic medical records: a review. *Journal of Healthcare Engineering*.

[46] Gong L. J., Zhang Z. F., Chen S. Q. (2020). Clinical named entity recognition from Chinese electronic medical records based on deep learning pretraining. *Journal of Healthcare Engineering*.

